RETRACTED

# Preventive Effects of Mandarin Fruit Peel Hydroethanolic Extract, Hesperidin, and Quercetin on Acetaminophen-Induced Hepatonephrotoxicity in Wistar Rats

**DOI:** 10.1155/2022/7065845

**Published:** 2022-09-02

**Authors:** Doaa Nor Eldin, Hanaa I. Fahim, Heba Y. Ahmed, Mohamed A. Abdelgawad, Mohammed A. S. Abourehab, Osama M. Ahmed

**Affiliations:** ^1^Physiology Division, Zoology Department, Faculty of Science, Beni-Suef University, P.O. Box 62521, Beni-Suef, Egypt; ^2^Rodents Division, Department of Harmful Animals, Plant Protection Research Institute, Agriculture Research Center, Egypt; ^3^Department of Pharmaceutical Chemistry, College of Pharmacy, Jouf University, Sakaka, Al Jouf 72341, Saudi Arabia; ^4^Department of Pharmaceutics, College of Pharmacy, Umm Al-Qura University, Makkah 21955, Saudi Arabia; ^5^Department of Pharmaceutics and Industrial Pharmacy, Faculty of Pharmacy, Minia University, Minya 61519, Egypt

## Abstract

Acetaminophen, also known as N-acetyl-para-aminophenol (NAPAP), is a traditional antipyretic and analgesic that is used extensively around the world to treat colds and fevers. However, a NAPAP excess causes rapid, severe liver and kidney damage. The goal of the study was to examine the protective effects and determine the mechanisms of action of MPHE, hesperidin, and quercetin in NAPAP-induced hepatorenal damage in Wistar rats. Male Wistar rats received a 0.5 g/kg oral supplement of NAPAP every other day for a period of four weeks. During the same period of NAPAP supplementation, MPHE (50 mg/kg), quercetin (20 mg/kg), and hesperidin (20 mg/kg) were administered to rats receiving NAPAP. MPHE, quercetin, and hesperidin treatments significantly improved liver function in NAPAP-supplemented rats. The high serum levels of aminotransferases, alkaline phosphatase, lactate dehydrogenase, and *γ*-glutamyl transferase as well as total bilirubin were significantly reduced, while the levels of suppressed serum albumin were significantly increased, demonstrating this improvement. Treatments utilizing these natural substances significantly enhanced kidney function as seen by a considerable decline in the increased blood levels of urea, uric acid, and creatinine. Additionally, the injection of MPHE, hesperidin, and quercetin resulted in a decrease in the quantity of lipid peroxides while increasing the activities of superoxide dismutase, glutathione peroxidase, and glutathione-S-transferase in the liver and kidneys. The treatments markedly abated the NAPAP-induced liver and kidney histological perturbations and reduced the NAPAP-induced serum tumor necrosis factor-*α* level and liver and kidney proapoptotic protein 53 and caspase 3 expressions. Otherwise, serum interleukin-4 level significantly increased by treatments. The MPHE, hesperidin, and quercetin treatments resulted in marked decrease in liver and kidney histopathological scores including inflammation, necrosis, apoptosis, and congestion. In conclusion, the MPHE, quercetin, and hesperidin may induce hepatonephropreventive impacts in NAPAP-supplemented rats *via* enhancing the antioxidant defense system, anti-inflammatory activity, and antiapoptotic action.

RETRACTED

## 1. Introduction

The liver is a substantial organ, which directs various essential metabolic capacities, maintains homeostatic condition in the body, and has an important function in detoxifications of xenobiotics, common toxins, and chemotherapeutic operators [1–3]. Exposure to various xenobiotics, which is a significant risk factor for many illnesses, has been viewed as a significant public health concern [4]. Foreign chemicals include environmental pollutants, toxicants, food additives, colorants in the pharmaceutical industries, and drugs, such as paracetamol, ibuprofen, doxorubicin and aminoglycosides [5–11]. Such chemicals and drugs often accumulate within the body and cause metabolic alkalosis, brain dysfunctions, cardiac arrhythmias, and hepatorenotoxicities [12, 13]. Hepatotoxicity is a general term for liver damage and is often an adverse side effect of long-term administration of many drugs that enter the liver through the hepatic portal vein and are subjected to the 1^st^ path of metabolism in the liver. The lesions due to hepatotoxicity may include necrosis, steatosis, fibrosis, cholestasis, and vascular injury [14]. Nephrotoxicity is a result of deficiency in kidney detoxification and excretion due to devastation of kidney function by toxicants [4].

Acetaminophen, also known as N-acetyl-para-aminophenol (NAPAP), paracetamol, and other over-the-counter antipyretic and analgesic medications can be harmful to the liver and kidneys when used over an extended period of time [15, 16]. N-Acetyl-P-benzoquinone imine (NAPQI), which is formed when the liver's cytochrome P450 (CYP450) system is activated at hazardous dosages, is the main reactive metabolite of NAPAP [17]. This compound causes hepatotoxicity and nephrotoxicity by reducing liver glutathione (GSH) concentration by 80–90% and binding covalently to protein and other macromolecules [18].

Plants play an essential role in human foods and medication. The nutritional treatment has recently been suggested in international literature. The use of natural plants as food and for phytotherapy to improve health and prevent and treat illnesses is a relatively new idea [19, 20]. Common antioxidants called flavonoids are found in foods with a plant origin and have a wide range of biological effects on different mammalian cell systems both in vivo and in vitro [15, 16, 21]. Citrus fruit extracts are rich in flavonoids and have strong antifree radical effects [22–24]. Citrus fruits contain the active flavonoid hesperidin, which possesses anti-inflammatory and antioxidant properties [25].

RETRACTED

Citrus fruits including oranges, lemons, and grapefruits contain hesperidin (3,5,7-trihydroxy flavanone-7-rhamnoglucoside), a bioflavonoid with potent pharmacological effects [26]. Hesperidin contains lipid-lowering, antioxidant, anti-inflammatory, antihypertensive, anticarcinogenic, and antiedema capabilities [27]. It also exhibits hydrogen radical- and hydrogen peroxide-removal activities [28].

A second flavonoid of plant origin called quercetin may be found in fruits and vegetables. The primary function of quercetin is its antioxidant activity through the scavenging of reactive oxygen species (ROS) [24, 29, 30]; it also exhibits anti-inflammatory and antifibrotic activities [31–33].

Therefore, the study aim was to assess the efficacies and modes of actions of mandarin (*Citrus reticulata* L.) fruit peel hydroethanolic extract (MPHE), quercetin, and hesperidin in NAPAP-induced hepatotoxicity and nephrotoxicity in Wistar rats.

## 2. Material and Methods

### 2.1. Experimental Animals and Housing

The National Research Center (NRC), Cairo, Egypt, provided the Wistar male rats used in this study, which weighed 130-150 g and were 10-12 weeks old. The rats were housed in well-ventilated cages at the Animal House of the Faculty of Science at Beni-Suef University, Egypt, between 20°C and 25°C with a 12-hour daily light/12-hour dark cycle. In addition to a daily normal pelleted food, the rats received unlimited access to water. The animals were held for 15 days before the start of the experiment to eliminate any current infections. All of the research was conducted in accordance with the regulations established by the Faculty of Science's Experimental Animals Ethics Committee at Beni-Suef University in Egypt (Ethical Approval Number BSU/FS/2014/11).

### 2.2. Chemicals

From Sigma-Aldrich (St. Louis, MO, USA), NAPAP, hesperidin, and quercetin were obtained. All other compounds utilized in this project were of the highest purity or analytical quality.

### 2.3. Preparation of Mandarin Fruit Peel Hydroethanolic Extract (MPHE)

Mandarin fruits had been bought from local markets in the Beni-Suef Governorate, Egypt, and were authenticated by staff members of Plant Taxonomy, Department of Botany, Faculty of Science, Beni-Suef University, Egypt. To guarantee that any dusts or pollution was removed, mandarin oranges were washed multiple times in tap water and then in distilled water (dist. water). The peels were allowed to dry for 20 days in a shaded, ventilated location. The dried peels were roughly crushed into a powder and left to soak in 70% ethanol for three days. The suspensions were frequently stirred.

RETRACTED

After filtering the hydroethanolic extract via Whatman filter paper, it was evaporated on a rotary evaporator with decreased pressure to produce the viscous residue, which was the MPHE [15, 23, 30, 34]. The MPHE, hesperidin, and quercetin dosages were dissolved in 1% carboxymethylcellulose (CMC).

### 2.4. Animal Grouping

The rats used in this experiment were divided into five groups (six for each) as follows (Figure 1):

Group 1 (normal control group): healthy normal rats were given the equivalent volume (5 ml/kg b.w.) of distilled water (a vehicle for NAPAP) and 1% CMC (a vehicle for MPHE, hesperidin, and quercetin) every other day per os (by mouth, orally) for 4 weeks.

Group 2 (NAPAP group): every other day for 4 weeks, 0.5 g/kg b.w. of NAPAP (dissolved in distilled water) was administered per os [15, 23, 35]. Additionally, throughout the same duration, the rats in this group received an equivalent volume of 1 percent CMC (5 ml/kg b.w.) every other day.

Group 3 (NAPAP+MPHE group): NAPAP was administered per os as in group 2. The rats were also treated with MPHE at 50 mg/kg b.w. [34] every other day per os for 4 weeks.

Group 4 (NAPAP+hesperidin group): NAPAP was administered per os as in group 2. The rats were also treated with hesperidin at 20 mg/kg b.w. [36] per os every other day for 4 weeks.

Group 5 (NAPAP+quercetin group): NAPAP was administered per os as in group 2. The rats were also treated with quercetin at 20 mg/kg b.w. [37] every other day per os for 4 weeks.

### 2.5. Blood and Tissue Sampling

After 4 weeks, blood from the jugular veins of anaesthetized rats was taken, allowed to coagulate, and then centrifuged for 15 minutes at 3000 rpm at room temperature (22°C). The sera were quickly separated and stored at -30°C in a deep freezer pending the discovery of several biochemical tests relating to liver and kidney function.

The rats were dissected after having their blood sampled. Each rat's longitudinal half of the kidney and pieces of the liver (5 mm^3^) were fixed in 10 percent neutral buffered formalin for histological research. Another 0.5 g of the liver and 0.5 g of the kidney of each rat were separately homogenized in 5 ml of 0.9% NaCl. The homogenate from each sample was centrifuged for 15 minutes at 3000 rpm. The supernatants were fractionated into three vials, aspirated, and stored at -30°C in a deep freezer to identify oxidative stress and antioxidant markers.

RETRACTED

### 2.6. Determination of Serum Biomarkers Related to Liver Function

Based on the methodologies of Bergmeyer et al. [38] and Gella et al. [39], Schumann et al. [40], and Szasz et al. [41], the serum alanine aminotransferase (ALAT) and aspartate aminotransferase (ASAT), alkaline phosphatase (AP), and *γ*-glutamyl transferase (*γ*GT) activities were examined using reagent kits purchased from Biosystem S.A. (Spain). Using reagent kits acquired from Spinreact (Spain), lactate dehydrogenase (LDH) activity was found using the method of Pesce [42]. HUMAN Gesellschaft für Biochemica und Diagnostica mbH, Wiesbaden, Germany, provided the kits used to measure albumin and total bilirubin levels based on the protocols of Doumas et al. [43] and Jendrassik and Grof [44], respectively.

### 2.7. Detection of Kidney Function Biomarkers in Serum

Serum creatinine and urea levels were tested in accordance with the guidelines of Fabiny and Ertingshausen [45] and Tabacco et al. [46] using reagent kits provided by Biosystem S.A. (Spain). The serum level of uric acid was determined using tools supplied by Spinreact (Spain) using an enzymatic colorimetric technique based on the technique published by Fossati et al. [47].

### 2.8. Detection of Serum Tumor Necrosis Factor-*α* (TNF-*α*) and Interleukin-4 (IL-4) Levels

Using kits provided by R&D Systems (USA), the sandwich enzyme immunoassay was used to assess the concentrations of TNF-*α* and cytokine IL-4 in the serum. This method was based on the established principles and procedures of Howard and Harada [48] and Croft et al. [49].

### 2.9. Assay of Oxidative Stress and Antioxidant Biomarkers in the Liver and Kidney

Based on the technique developed by Beutler et al. [50], malondialdehyde (MDA) generation from hepatic and renal lipid peroxidation (LPO) was identified. Preuss et al.'s [51] technique was used to determine GSH content. Based on the methods and concepts of Matkovics et al. [52], Mannervik and Gutenberg [53], and S. Marklund and G. Marklund [54], the activities of glutathione peroxidase (GPx), glutathione-S-transferase (GST), and superoxide dismutase (SOD) in the liver and kidney were measured. All of the chemicals used to make the reagents for measuring oxidative stress and antioxidant parameters were of analytical quality.

### 2.10. Detection of Proapoptotic Protein 53 (p53) and Caspase 3 by Western Blotting

Caspase 3 and p53 of the liver and kidney were analyzed using western blotting. RIPA (radioimmunoprecipitation assay) buffer was used to homogenize liver and kidney samples, and the clear supernatant was obtained by centrifuging the mixture. The total protein content was determined using the Bradford reagent. SDS-PAGE was then used to separate 30 *μ*g of protein per gel lane, which was then transferred to a polyvinylidene difluoride (PVDF) membrane. After that, the membranes were treated with p53 (R&D Systems, Bio-Techne Brands, USA), caspase 3 (NSJ Bioreagents, San Diego, CA, USA), and *β*-actin primary antibodies (NSJ Bioreagents, San Diego, CA, USA). After that, the membranes were blocked with Tris-buffered saline containing Tween 20 (TBST) and 5 percent nonfat milk powder (Novus Biologicals, Littleton, CO, USA). As a loading control, the housekeeping protein *β*-actin was utilized to make sure that protein loading was equal throughout the gel and to standardize the quantities of protein identified. After being TBST-washed, the membranes were treated for an hour with Novus Biologicals' secondary antibodies (Novus Biologicals, Littleton, Colorado, USA) that were conjugated to horseradish peroxidase. Immunolabeling was developed using a kit with enhanced chemiluminescence (BioRad, Hercules, CA, USA). Following scanning of the resulting blots, band intensities were measured using ImageJ (NIH, Bethesda, Maryland, USA).

RETRACTED

### 2.11. Histological Investigations

The liver and kidneys from each rat were quickly removed after sacrifice, decapitation, and dissection, and then, they were perfused with saline solution. Pieces from the liver and the longitudinal half of one kidney of each rat were taken and fixed in 10% neutral buffered formalin for 24 hours. The steps for processing organ specimens for histological section preparation and hematoxylin and eosin (H&E) staining were carried out in accordance with the guidelines and procedures of Bancroft et al. [55]. The histologically stained liver and kidney sections were examined by a histopathologist to detect the histopathological lesions. The lesion scores were also detected and were graded 0, I, II, and III for the absence of lesion, mild, moderate, and severe, respectively.

### 2.12. Statistical Analysis

Data are represented using the mean and standard error of the mean (*M* ± SEM). The statistical analysis was performed using SPSS (Statistical Package for the Social Sciences; version 22) (IBM SPSS for Windows, IBM Corp., Armonk, NY). Tukey's post hoc test was used to compare mean values in pairs. Differences across groups were considered significant at *P* < 0.05.

## 3. Results

### 3.1. Effects on Serum Parameters Related to Liver Function

The effects of MPHE, hesperidin, and quercetin on serum ALAT, ASAT, AP, *γ*GT, and LDH activities as well as total bilirubin and albumin levels in NAPAP-administered rats are represented in Tables 1 and 2. Oral administration of NAPAP showed significant increases of 174.18%, 112.27%, 79.41%, 182.28%, and 98.31%, respectively, in serum ALAT, ASAT, AP, *γ*GT, and LDH activities relative to the activities in the normal control rats (*P* < 0.05) (Table 1). Treatment of the NAPAP-administered rats with MPHE decreased the elevated activities of ALAT, ASAT, AP, *γ*GT, and LDH by −64.9%, −44.40%, −53.27%, −68.01%, and −54.77%, respectively, relative to the activities in the NAPAP rats. Administration of hesperidin to the APAP-administered rats alleviated the adverse effects induced by NAPAP; the recorded percentage changes of ALAT, ASAT, AP, *γ*GT, and LDH decreased by −64.12%, −49.94%, −48.08%, −68.01%, and −51.98%, respectively, relative to the activities in the NAPAP rats. Hesperidin treatment decreased the increased levels of liver enzymes. For treatment with quercetin, the changes in ALAT, ASAT, AP, *γ*GT, and LDH activities were −62.92%, −47.82%, −55.05%, −66.26%, and −51.96%, respectively, relative to those of the NAPAP rats. The administration of NAPAP to normal rats significantly increased the serum total bilirubin level by 87.14% and depleted serum albumin content by −16.09% relative to those of normal rats (*P* < 0.05). On the other hand, the treatment of NAPAP-administered rats with MPHE, hesperidin, and quercetin ameliorated the total bilirubin levels significantly by −51.90%, −53.43%, and−48.85%, respectively, relative to those of NAPAP rats (*P* < 0.05). Additionally, these treatments induced increases in the decreased albumin level by 15.49%, 17.71%, and 19.18%, respectively (*P* < 0.05). MPHE administration was more potent in decreasing LDH activity. On the other hand, hesperidin was better at decreasing ASAT and total bilirubin levels. The effects on AP activity and albumin level were highest after quercetin administration. Moreover, the effect of MPHE and hesperidin was more or less similar on serum ALAT and *γ*GT activities.

RETRACTED

### 3.2. Effects on Serum Parameters Related to Kidney Function

The effects of MPHE, hesperidin, and quercetin on serum urea, uric acid, and creatinine levels of NAPAP-administered rats are shown in Table 3. The administration of NAPAP to normal rats elevated serum urea, uric acid, and creatinine levels by 168.24%, 92.59%, and 83.02%, respectively, relative to those in normal rats (*P* < 0.05). Treatment of NAPAP-administered rats with MPHE prevented increases in serum urea, uric acid, and creatinine levels by −62.72%, −55.13%, and−45.36%, respectively (*P* < 0.05). Additionally, oral supplementation of NAPAP-administered rats with hesperidin and quercetin reduced the elevated levels of serum urea, uric acid, and creatinine levels (*P* < 0.05). The recorded percentage changes of serum urea, uric acid, and creatinine levels were -55.93%, -56.41%, and -47.42%, respectively, due to treatment with hesperidin, while they were -59.81%, 59.94%, and -53.61%, respectively, due to treatment with quercetin. Treatment with a MPHE had the most potent effect in lowering serum urea level (−62.72%), whereas quercetin treatment was the most effective in decreasing the elevated uric acid and creatinine levels (−59.94% and −53.61%, respectively).

### 3.3. Influences on IL-4 and TNF-*α* Levels

The effects of MPHE, hesperidin, and quercetin on serum TNF-*α* and IL-4 concentrations of NAPAP-administered rats are shown in Table 4. Oral administration to normal rats with NAPAP led to a 295.60% increase (*P* < 0.05) in the serum proinflammatory cytokine TNF-*α* and a −67.82% decrease (*P* < 0.05) in the serum anti-inflammatory cytokine IL-4 relative to the levels in normal control rats. Treatment of NAPAP-administered rats with MPHE, hesperidin, and quercetin led to decreases in serum TNF-*α* of −24.11%, −30.95%, and−41.63%, respectively, relative to the levels in normal rats (*P* < 0.05). Conversely, the serum IL-4 level was increased by 136.14%, 128.75%, and 135.39%, respectively, relative to the levels in normal rats (*P* < 0.05).

### 3.4. Effects on Liver Oxidative Stress and Antioxidants

Data showing the effects of MPHE, hesperidin, and quercetin on liver SOD and LPO levels in NAPAP-administered rats are presented in Table 5. The administration of NAPAP to normal rats produced a significant increase (*P* < 0.05) in LPO level by 113.10%, whereas liver SOD activity significantly decreased by −34.55%. The treatment of NAPAP-administered rats with MPHE, hesperidin, and quercetin ameliorated the increased LPO level greatly by −37.20%, −31.30%, and−24.44%, respectively (*P* < 0.05). The treatment of NAPAP-administered rats with MPHE, hesperidin, and quercetin increased the decreased SOD activity by 45.75%, 36.30%, and 39.45%, respectively (*P* < 0.05). MPHE showed the most potent effect in increasing SOD level and decreasing LPO level. Treatments of the NAPAP-administered rats with the three tested natural products alleviated the lowered levels of liver GPx, GSH, and GST. Quercetin treatment showed the most potent effect on the three antioxidant enzymes.

### 3.5. Effects on Kidney Oxidative Stress and Antioxidants

Table 6 shows the effects of MPHE, hesperidin, and quercetin on kidney LPO and GSH content and GST, GPx, and SOD activities of the NAPAP-administered rats. NAPAP administration decreased GSH content and GPx, GST, and SOD activities relative to those of the normal control group by −31.86%, −6.60%, −18.07%, and −21.35%, respectively (*P* < 0.05). On the other hand, administration of NAPAP to normal rats increased LPO level by 53.35% relative to that in the controls (*P* < 0.05). MPHE ameliorated the decrease in GSH content (*P* < 0.05) and in GPx (*P* < 0.05), GST (*P* < 0.05), and SOD activities by 33.52%, 4.56%, 13.31%, and 0.59%, respectively, relative to those in normal rats. Additionally, this extract diminished the increase in LPO level greatly by −26.04% (*P* < 0.05). Oral treatment of hesperidin to NAPAP-administered rats improved the lowered GSH content and GPx, GST, and SOD activities by 29.88%, 5.15%, 15.02%, and 10.64%, respectively (*P* < 0.05). The elevated LPO level decreased by −19.24% relative to that in the controls (*P* < 0.05). Treatment of NAPAP-administered rats with quercetin improved the lowered GSH content and GPx, GST, and SOD activities by 35.29%, 4.70%, 12.59%, and 19.85%, respectively (*P* < 0.05). The LPO level decreased after quercetin administration. Treatment with quercetin showed the most potent effect in increasing GSH and SOD levels, whereas treatment with hesperidin was most effective in increasing GST and GPx. The MPHE had the most potent effect in decreasing LPO level.

RETRACTED

### 3.6. Effect on Caspase 3 Protein Expression in the Liver and Kidney

The expression protein levels of liver and kidney proapoptotic mediators p53 and caspase 3 are depicted in Figures 2 and 3. The NAPAP-administered rats exhibited a significant increase (*P* < 0.05) in both liver and kidney p53 and caspase 3 levels. The treatment with MPHE, hesperidin, and quercetin significantly reduced (*P* < 0.05) the NAPAP-induced increases in p53 and caspase 3 protein expressions in both the liver and kidney. While the improvement effect of hesperidin was the most potent on liver p53, the quercetin was the most effective in downregulating the higher kidney p53 and caspase 3 expression levels.

### 3.7. Histopathological Changes

#### 3.7.1. Liver

Normal histoarchitecture of the central vein, hepatocytes, and hepatic sinusoids was seen in the liver sections of healthy rats (Figure 4(a)). Following the administration of NAPAP, the liver underwent a number of lesions and histological changes, including cytoplasmic vacuolizations of hepatocytes, focal hepatic necrosis associated with inflammatory cell infiltration, a large number of apoptotic cells, portal infiltration with mononuclear leucocytic inflammatory cells, and congestion of the central vein (Figures 4(b)–4(d)). When rats receiving NAPAP were given MPHE, the hepatic tissue underwent alterations that included mild sinusoidal leukocytosis, cytoplasmic vacuolizations of hepatocytes, Kupffer cell activation, a small number of apoptotic cells, and slight sinusoidal congestion (Figures 5(a) and 5(b)). Additionally, the treatment with hesperidin resulted in cytoplasmic vacuolizations of hepatocytes, few apoptotic cells, and congestions of the central veins (Figures 5(c) and 5(d)). When quercetin was given to rats receiving NAPAP, it caused minor sinusoidal congestions, a small number of inflammatory cells, activated Kupffer cells, and apoptotic bodies (Figures 5(e) and 5(f)).

RETRACTED

Liver histopathological scores of study groups were represented (Table 7). Rats under normal management did not have any histological lesions in their liver sections, scoring 0 points. The liver histological lesions, such as inflammation, necrosis, activated apoptosis, cytoplasmic vacuolizations of hepatocytes, vascular congestion, and Kupffer cells' proliferation (activation), significantly improved after MPHE, hesperidin, and quercetin treatments were given to rats that had received NAPAP. Most of the treated rats showed lower grades of lesion scores than the NAPAP-administered rats.

#### 3.7.2. Kidney

The histopathological findings showed normal kidney architecture in the control group (Figure 6(a)), in contrast to the NAPAP-administered group, and congestions of renal blood vessels, apoptotic cells, and focal necrosis of renal tubules accompanied by inflammatory cell infiltrations were observed, which were indications of renal damage (Figures 6(b) and 6(c)). Treatment of NAPAP-administered rats with the MPHE showed improvement of the kidney histological structure, which attained its normal structure (Figures 7(a) and 7(b)). Administration of hesperidin induced ameliorative effects in kidney sections with slight vacuolation of the renal tubular epithelium (Figures 7(c) and 7(d)). Treatment of NAPAP-administered rats with quercetin alleviated adverse effects in kidney sections, but slight congestion of the glomerulus was noted (Figures 7(e) and 7(f)).

Table 8 shows the kidney histopathological scores of study groups. Rats under normal control conditions' kidney sections showed no histological lesions, resulting in a score of 0. The kidney histological lesions, including inflammation, necrosis, apoptosis, and vascular congestion, remarkably improved when NAPAP-administered rats received treatments with MPHE, hesperidin, and quercetin. Most treated rats showed lower grades of lesion scores than NAPAP-administered rats.

## 4. Discussion

NAPAP, an over-the-counter medication, looks to be a safe and effective treatment for pain, fever, and inflammation when used as directed [56, 57]. NAPQI, a hazardous metabolite produced by CYP450 in response to drug overdoses, can cause immediate liver and kidney damage [58–60]. NAPAP is metabolized in the liver, with the hepatic CYP450 system being responsible for 5–10% of the process. Besides sulfation and glucuronidation, the glutathione redox system plays a crucial part in neutralizing the metabolite produced by glutathione conjugation, which depletes the liver's supply of GSH. The rapid transformation of NAPAP into the reactive metabolite NAPQI by CYP450 enzymes, namely, cytochrome P450 family 2 subfamily E member 1 (CYP2E1), impacts the generation of free radicals that, when covalently bound to cellular nucleophiles such DNA, RNA, and proteins, cause cell damage [61, 62]. Thus, the NAPAP (acetaminophen) toxicities are mainly due to the elevated levels of NAPQI that result in depletion of GSH leading to less scavenging of free radicals and ROS [63–66]. Considering this attribution, the use of natural antioxidants such as plant extracts and constituents such as flavonoids as an antidote against an APAP overdose may be applicable to abate APAP toxicity.

RETRACTED

Hepatic cells contain a group of enzymes that have been used as markers for recognizing liver damage. ALAT, ASAT, and AP levels are elevated in blood following liver cell damage [67]. In the current study, NAPAP oral administration in a dose level of 0.5 g/kg every other day for four weeks increased serum transaminase, LDH and *γ*GT activities, and bilirubin level relative to those in the normal control group; these recorded effects are consistent with those in past reports [14, 68–70]. The serum or plasma ASAT levels may rise as a result of muscle injury, myocardial infarction, and viral hepatitis. ASAT is released in a similar way and catalyzes the conversion of alanine to pyruvate and glutamate. On the other hand, ALAT is more specific to the liver and thereby is a primary factor related to liver damage. It has been demonstrated that the liver's increased hepatic enzyme activity is linked to cellular leakage and a loss of cell membrane functional integrity [1, 71]. ASAT, ALAT, and LDH enzymes are cytosolic enzymes of hepatocytes, and increases in these enzyme activities in NAPAP-administered rats are due to their increased leakage from necrotic hepatocytes [72, 73]. The rise of AP and GT, two membrane-bound enzymes, may be brought on by an increased rate of synthesis and/or regurgitation into the blood as a result of bile ductule occlusion [72]. Hepatobiliary disease was verified by the rise in AP and GT activities in conjunction with the elevation in blood total bilirubin levels [74]. According to previous publications, the pathological modification in biliary flow is what causes the rise in AP and bilirubin levels in animals treated with NAPAP [75]. It is also important to note that hyperbilirubinemia has been linked to unconjugated and conjugated bilirubin release from injured hepatocytes, increased heme degradation, occlusion of hepatic bile ducts, and inhibition of the conjugation response [76]. Along with ALAT and ASAT, the cytoplasmic enzyme LDH is also elevated NAPAP administration. Nicotinamide adenine dinucleotide (NADH) is converted from its reduced form to its oxidized form, nicotinamide adenine dinucleotide (NAD^+^), concomitant with the conversion of pyruvate to lactate *via* the action of the enzyme LDH [77]. The increase in LDH activity could be explained by cellular injury causing the enzyme to seep from tissues into the blood. In this investigation, delivery of NAPAP resulted in a substantial rise in serum LDH. Similar outcomes were attained by Farghaly and Hussein [78] who observed that oral treatment of NAPAP (500 mg/kg) induced a substantial rise in serum LDH compared to those in normal rats. The acquired results are in agreement with those of Lebda et al. [79] who reported that LDH in NAPAP-medicated rats was critically raised during a 21-day investigation. The intracellular accumulation of calcium ion (Ca^2+^), which triggers phosphofructokinase and anaerobic glycolysis-enhancing lactate production, may be the reason of the increase in cytosolic LDH activity by NAPAP [80]. In the case of NAPAP, the process of cell death may reach an irreversible final stage in which Ca^2+^ homeostasis is lost as a result of oxidative damage and an increase in intracellular Ca^2+^ [81]. The current data are compatible with those of Abd El Fadil et al. [82] who demonstrated that NAPAP promoted toxic damage to rat hepatic cells as indicated by a critical increase in LDH leakage. In contrast to the pattern of serum total bilirubin level, the results of a research by Okokon et al. [83] show that NAPAP-administered rats had significantly lower blood albumin levels. This drop in albumin levels in rats receiving NAPAP may be brought about by necrosis, apoptosis, and liver cell degeneration, which result in a reduction in the number of cells producing albumin [84].

RETRACTED

Histological findings showing the presence of cytoplasmic vacuolization of hepatocytes, focal hepatic necrosis associated with inflammatory cell infiltration, numerous apoptotic cells, portal infiltration with inflammatory cells, and congestion of the central vein support the impairment in liver function parameters in serum, including ALAT, ASAT, AP, GT, and LDH activities, as well as total bilirubin and albumin levels, caused by NAPAP administration.

In our investigation, administration of the MPHE considerably increased the serum activity of hepatic enzymes. In line with the present findings, earlier research [34] showed the hepatoprotective efficacy of mandarin extract against NAPAP overdose-induced hepatocyte injury in male rats. Citrus byproduct extracts' ability to protect the liver may be due to the presence of phytoconstituents like phenolic compounds, particularly the distinctive flavanones, which are mostly composed of naringin, hesperidin, narirutin, and neohesperidin [14, 85, 86]. In the present study, supplying quercetin and hesperidin to NAPAP-supplemented rats markedly diminished serum levels of ALAT, ASAT, AP, LDH, and *γ*GT activities and bilirubin concentration together with a significant increase in serum albumin level, suggesting that quercetin and hesperidin possess hepatoprotective activity that could be attributed to the antioxidant potencies of quercetin and hesperidin [87]. The current histological results support this possibility since oral administration of MPHE, hesperidin, and quercetin induced remarkable amelioration of the liver tissue devastated by NAPAP administration.

Oral administration of NAPAP in this study prompted renal damage evidenced by the elevation in serum concentrations of creatinine, urea, and uric acid. These data agree with those of other publications [14, 88, 89]. Urea is a byproduct of protein metabolism, and its increase is an important marker of renal toxicity [16]. Additionally, increases in creatinine concentration are related to glomerular function and indicate renal failure [90]. Serum uric acid concentrations have been supposed as one of the potential risk factors for renal disease's potential development [91]. According to Ajami et al. [92] and Ahmed et al. [14], oxidative stress and renal damage are strongly correlated, which may explain why serum creatinine, urea, and uric acid levels increased following NAPAP treatment. High ROS generation may modify the filtration coefficient and alter the filtration surface area, which may reduce glomerular filtration and lead to the buildup of urea and creatinine. This study demonstrated obvious histopathological alterations of the kidney, confirming that NAPAP induced kidney injury. These histological changes include interstitial nephritis, localized necrosis of the renal tubules, congested glomerular tuft and renal blood vessels, and many apoptotic cells. In our investigation, MPHE significantly reduced the raised serum levels of kidney function indices, such as creatinine, urea, and uric acid, and enhanced kidney histological architecture and integrity in the rats that had been given NAPAP. Our findings are consistent with Ahmad et al. [93] and Mostafa et al. [34]. The inclusion of flavonoids in the citrus extract may be the cause of MPHE's powerful effects. Mandarin offers nutritional value because of its unique makeup. Citrus pulp and peel have been shown to contain flavonoids, particularly polymethoxy flavones and flavones (hesperidin, narirutin, and naringin) [94]. The peel of this citrus also has many biological properties due to high concentrations of flavonoids [95]. An extract from the fruit of a *Citrus reticulata* cv. Chachiensis is abundant in bioactive substances, such as ascorbic acid and carotenoids, but because it contains less sugar than other types and hence has a lower acidic content, it cannot compete in the market for citrus juice [96]. Additionally, in the current study, quercetin and hesperidin treatment of NAPAP-administered rats resulted in significantly lower serum levels of creatinine, urea, and uric acid, suggesting nephroprotective activity of quercetin and hesperidin that may be attributed to their potential antioxidant activities [87, 97]. These effects have been correlated with the ameliorative effects shown in kidney tissues in treated groups.

RETRACTED

The inevitable byproducts of oxidative metabolic activities, or ROS, lead to oxidative stress and cell damage that can be reduced by antioxidants [98]. Finding reliable and potent antioxidants is therefore crucial. The potential of natural compounds, such as phenols and flavonoids, to heal liver damage has reportedly been linked to their antioxidant activity [99–102].

An increase in hepatic and renal LPO and a reduction in GSH content, as well as GPx, GST, and SOD activities, were both significantly induced by NAPAP administration in the current investigation, which encouraged disturbance of the oxidant/antioxidant state. These results are consistent with those from other publications [14, 16, 23, 103]. The hazardous metabolite NAPQI, a byproduct of NAPAP that has a strong affinity for GSH and depletes it, may accumulate as a result of the enhanced oxidative stress, at least in part [104]. By disrupting the bilayer structure and changing membrane characteristics such fluidity, permeability to various substances, bilayer thickness, and triggering membrane, LPO has an effect on the liver [105, 106]. The elevation in the MDA level is an indicator of LPO [106]. Overproduction of free radicals and ROS during NAPAP metabolism causes a drain of the natural body antioxidant system and promotes LPO, as evidenced by an observed diminishment in the level of SOD and GPx and rise of MDA content in a previous study [82]. The elevation in liver MDA production by NAPAP reported in our trials is consistent with the increases in previous studies, which reported that NAPAP elevated extracellular MDA level [107]. Elevation of LPO may result in damage to biologically important molecules and tissues [108].

RETRACTED

The present results explore that administration of MPHE, hesperidin, and quercetin increased antioxidant (GSH, GST, SOD, and GPx) levels and depleted oxidant (MDA) level relative to those in the NAPAP-administered rats. SOD transforms superoxide anion O_2_^·^ to hydrogen peroxide. GPx catalyzes decreases in hydrogen peroxide and other peroxides by coupling with GSH [109, 110]. Citrus fruit peels are recognized to have antibacterial, anticancer, anti-inflammatory, and antioxidant properties [111–114], so the treatment of NAPAP-administered rats with MPHE for 4 weeks in our study induced a hepato-renal protective effect marked by enhanced activities of hepatic and renal enzymes and concentrations of albumin and bilirubin in serum in coordination to the ameliorative effects on the redox status of the tissues. These data are concordant with results of Ahmad et al.'s [93] and Mostafa et al.'s [34] publications. The bioactive constituents in MPHE as flavonoids, phenolics, and steroids [86] may play a crucial role in changing hepatorenal function and the antioxidant defense system. The protective potentials of flavonoids in biological systems are attributed to their ability to inhibit oxidative stress and LPO [115, 116].

In terms of the impact on inflammation, oral administration of NAPAP markedly elevated the blood levels of the proinflammatory cytokine TNF-*α* and lowered the levels of the anti-inflammatory interleukin IL-4. These pieces of information agree with those of Ahmed et al. [14]. TNF-*α* is known to draw in and energize more inflammatory cells [117] and has been associated with increased oxidative stress [117]. Several studies have stated that NAPAP-induced liver injury might be promoted by stimulating the oxidative stress and the inflammatory response [14, 118–120]. Attenuation of NAPAP-mediated liver damage was able to be obtained by repressing inflammatory and proinflammatory cytokine release, *viz*, TNF-*α* and IL-6 [121, 122]. The treatment of NAPAP-supplied rats with MPHE, hesperidin, and quercetin in the present study improved the higher TNF-*α* and lower IL-4 levels.

Concerning apoptosis, the proapoptotic proteins p53 and caspase 3 were detected in both the liver and kidney. In the present study, both proteins increased significantly in NAPAP-administered rats and the treatment with MPHE, hesperidin, and quercetin significantly reduced these NAPAP-induced elevations reflecting the antiapoptotic effects of MPHE, hesperidin, and quercetin (Figure 8). It is worth mentioning that p53 is an important mediator of intrinsic apoptosis [123, 124], and the activation of caspase 3 can be mediated by stimulation of both intrinsic and extrinsic pathways of apoptosis [36]. Moreover, TNF-*α* may activate the extrinsic pathway by binding to tumor necrosis factor receptors (TNFR) on the cell membrane [36] (Figure 8). Thus, according to the findings of the presented study and previous elucidations, it is suggested that MPHE, hesperidin, and quercetin have antiapoptotic actions which could be mediated *via* suppression of both intrinsic and extrinsic pathways of apoptosis (Figure 8).

RETRACTED

Taken together, this study showed that MPHE, hesperidin, and quercetin had hepatorenal preventive potentials by their abating impacts on oxidative stress, inflammation, and apoptosis (Figure 8).

## Figures and Tables

**Figure 1:** Diagram illustrating the experimental setup and animal grouping.

**Figure 2:** Effect of MPHE, hesperidin, and quercetin on liver p53 and caspase 3 expression levels in NAPAP-administered rats. (a) Immunoblots of liver p53, caspase 3, and *β*-actin. ^a^Significant at *P* < 0.05 in comparison with the normal values. ^b^Significant at *P* < 0.05 in comparison with NAPAP values.

**Figure 3:** Effect of MPHE, hesperidin, and quercetin on kidney p53 and caspase 3 expression levels in NAPAP-administered rats. (a) Immunoblots of kidney p53, caspase 3, and *β*-actin. ^a^Significant at *P* < 0.05 in comparison with the normal values. ^b^Significant at *P* < 0.05 in comparison with NAPAP values.

**Figure 4:** Photomicrograph of H&E-stained liver sections of normal and NAPAP-supplied rats: (a) normal liver section showing normal hepatocytes (H), sinusoid (S), and central vein (CV); (b) liver section of NAPAP-administered rats showing cytoplasmic vacuolization of hepatocytes (V), apoptotic cells (AC), and congestion of the central vein (C) accompanied by inflammatory cell infiltrations (IF); (c) liver section of NAPAP-administered rats showing cytoplasmic vacuolizations of hepatocytes (V), apoptotic cells (AC), and portal infiltration with inflammatory cells (IF); (d, e) liver section of NAPAP-administered rats showing cytoplasmic vacuolizations of hepatocytes (V), apoptotic cells (AC), and focal necrosis of hepatocytes (NC) accompanied by inflammatory cell infiltrations (IF). ×400.

**Figure 5:** Photomicrograph of H&E-stained liver sections of NAPAP-administered rats treated with MPHE (a, b), hesperidin (c, d), and quercetin (e, f): (a) liver section showing slight sinusoidal leukocytosis (SL) and Kupffer cell activation (KF); (b) liver section depicting slight cytoplasmic vacuolizations of hepatocytes (V), apoptotic cells (AC), and slight congestion of sinusoids (CS); (c) liver section showing cytoplasmic vacuolization of hepatocytes (V); (d) liver section showing cytoplasmic vacuolizations of hepatocytes (V), apoptotic cells (AC), and congestion of the central vein (C); (e) liver section showing Kupffer cell activation (KF), apoptotic bodies (AB), and congestion of hepatic sinusoids (CS) accompanied by few inflammatory cells; (f) liver section showing Kupffer cell activation (KF). ×400.

RETRACTED

**Figure 6:** Photomicrographs of kidney sections from NAPAP-administered rats and normal rats with H&E staining. Section through the kidney of a healthy rat is shown in (a). The glomerulus (G), proximal tubules (PT), and distal tubules are all healthy (DT). (b, c) NAPAP-administered rats had kidney sections that showed apoptotic cells and clogged renal blood channels (C) in (b) and apoptotic cells (AC) and focal necrosis of renal tubules (NC) accompanied by inflammatory cell infiltrations (IF) in (c). ×400.

**Figure 7:** Photomicrograph of H&E-stained kidney sections of NAPAP-administered rats treated with MPHE (a, b), hesperidin (c, d), and quercetin (e, f): (a, b) sections of the kidney showing no pathological changes; (c) section of the kidney showing apoptotic cell (AC) and slight vacuolations of the renal tubular epithelium (V); (d) section of the kidney showing no pathological changes; (e) section of the kidney showing slight congestion of the glomerulus (C); (f) section of the kidney showing no pathological changes. ×400.

**Figure 8:** Schematic figure showing the suggested mechanisms of action of MPHE, hesperidin, and quercetin in NAPAP-administered rats in light of the results of the current study.

**Table 1:** Effect of MPHE, hesperidin, and quercetin on serum ALAT, ASAT, AP, and *γ*GT activities of NAPAP-administered rats.

Groups	Parameter							
	ALAT (U/L)	% change	ASAT (U/L)	% change	AP (U/L)	% change	*γ*GT (mU/dl)	% change
Normal	30.33 ± 0.91		66.66 ± 1.54		408 ± 6.16		3.51 ± 0.42	
NAPAP	83.16 ± 1.16^a^	174.18	141.50 ± 2.59^a^	112.27	732 ± 6.94^a^	79.41	9.88 ± 0.31^a^	182.28
NAPAP+MPHE	29.16 ± 0.60^b^	-64.93	78.66 ± 1.72^b^	-44.40	342 ± 8.24^b^	-53.27	3.16 ± 0.30^b^	-68.01
NAPAP+hesperidin	29.83 ± 0.87^b^	-64.12	70.83 ± 1.83^c^	-49.94	380 ± 6.63^c^	-48.08	3.16 ± 0.30^b^	-68.01
NAPAP+quercetin	30.83 ± 0.79^b^	-62.92	73.83 ± 1.32^bc^	-47.82	329 ± 7.64^b^	-55.05	3.33 ± 0.21^b^	-66.26

Data are expressed as mean ± SEM. The number of animals in each group is 6. ^a^Significant at *P* < 0.05 in comparison with the normal values. ^b^Significant at *P* < 0.05 in comparison with NAPAP values. ^c^Significant at *P* < 0.05 in comparison with NAPAP+MPHE values. Percentage changes are calculated by comparing NAPAP-administered control with normal control and NAPAP-administered treated rats with NAPAP-administered control.

RETRACTED

**Table 2:** Effects of MPHE, hesperidin, and quercetin on serum total bilirubin and albumin levels and LDH activity of NAPAP-administrated rats.

Groups	Parameter					
	LDH (U/L)	% change	Total bilirubin (mg/dl)	% change	Albumin (g/dl)	% change
Normal	1776 ± 42.56		0.70 ± 0.04		3.23 ± 0.08	
NAPAP	3522 ± 98.20^a^	98.31	1.31 ± 0.12^a^	87.14	2.71 ± 0.07^a^	-16.09
NAPAP+MPHE	1593 ± 75.98^b^	-54.77	0.63 ± 0.01^b^	-51.90	3.13 ± 0.06^b^	15.49
NAPAP+hesperidin	1691 ± 69.45^b^	-51.98	0.61 ± 0.01^b^	-53.43	3.19 ± 0.07^b^	17.71
NAPAP+quercetin	1699 ± 71.56^b^	-51.96	0.67 ± 0.008^b^	-48.85	3.23 ± 0.12^b^	19.18

Data are expressed as mean ± SEM. The number of animals in each group is 6. ^a^Significant at *P* < 0.05 in comparison with the normal values. ^b^Significant at *P* < 0.05 in comparison with NAPAP values. Percentage changes are calculated by comparing NAPAP-administered control with normal control and NAPAP-administered treated rats with NAPAP-administered control.

**Table 3:** Effect of MPHE, hesperidin, and quercetin on serum urea, uric acid, and creatinine levels of NAPAP-administered rats.

Groups	Parameter					
	Urea (mg/dl)	% change	Uric acid (mg/dl)	% change	Creatinine (mg/l)	% change
Normal	25.66 ± 1.49		1.62 ± 0.14		0.53 ± 0.042	
NAPAP	68.83 ± 1.01^a^	168.24	3.12 ± 0.10^a^	92.59	0.97 ± 0.030^a^	83.02
NAPAP+MPHE	25.66 ± 1.11^b^	-62.72	1.40 ± 0.12^b^	-55.13	0.53 ± 0.042^b^	-45.36
NAPAP+hesperidin	30.33 ± 2.21^b^	-55.93	1.36 ± 0.07^b^	-56.41	0.51 ± 0.040^b^	-47.42
NAPAP+quercetin	27.66 ± 1.90^b^	-59.81	1.26 ± 0.07^b^	-59.94	0.45 ± 0.035^b^	-53.61

Data are expressed as mean ± SEM. The number of animals in each group is 6. ^a^Significant at *P* < 0.05 in comparison with the normal values. ^b^Significant at *P* < 0.05 in comparison with NAPAP values. Percentage changes are calculated by comparing NAPAP-administered control with normal control and NAPAP-administered treated rats with NAPAP-administered control.

**Table 4:** Effect of MPHE, hesperidin, and quercetin on serum TNF-*α* and IL-4 levels of NAPAP-administered rats.

Groups	Parameter			
	TNF-*α* (pg/ml)	% change	IL-4 (U/L)	% change
Normal	33.23 ± 1.56		122.63 ± 3.23	
NAPAP	131.46 ± 1.91^a^	295.60	40.23 ± 1.53^a^	-67.82
NAPAP+MPHE	99.76 ± 7.50^b^	-24.11	94.93 ± 5.54^b^	136.14
NAPAP+hesperidin	90.76 ± 5.95^bc^	-30.95	91.96 ± 7.99^b^	128.75
NAPAP+quercetin	76.73 ± 4.61^c^	-41.63	94.63 ± 3.08^b^	135.39

Data are expressed as mean ± SEM. The number of animals in each group is 6. ^a^Significant at *P* < 0.05 in comparison with the normal values. ^b^Significant at *P* < 0.05 in comparison with NAPAP values. ^c^Significant at *P* < 0.05 in comparison with NAPAP+MPHE values. Percentage changes are calculated by comparing NAPAP-administered control with normal control and NAPAP-administered treated rats with NAPAP-administered control.

RETRACTED

**Table 5:** Effect of MPHE, hesperidin, and quercetin in liver content of GSH and activities of GPx and GST and SOD and LPO in NAPAP-administered rats.

Parameter groups	LPO (nmole/100 mg tissue)	% change	SOD (U/g tissue)	% change	GSH (nmole/100 mg tissue)	% change	GPx (mU/100 mg tissue)	% change	GST (U/100 mg tissue)	% change
Normal	53.66 ± 1.11		99.55 ± 1.54		31.68 ± 0.67		185.26 ± 1.19		45.90 ± 1.34	
NAPAP	114.35 ± 1.28^a^	113.10	65.15 ± 2.92^a^	-34.55	20.81 ± 0.47^a^	-34.31	169.53 ± 2.37^a^	-8.49	34.05 ± 0.93^a^	-25.81
NAPAP+MPHE	71.81 ± 2.06^b^	-37.20	94.96 ± 1.48^bc^	45.75	29.43 ± 0.64^b^	41.42	181.83 ± 0.94^b^	7.25	41.23 ± 1.35^b^	21.08
NAPAP+hesperidin	78.55 ± 3.01^bc^	-31.30	88.80 ± 2.38^b^	36.30	29.88 ± 0.45^b^	43.58	181.85 ± 1.22^b^	7.26	42.06 ± 0.86^b^	23.52
NAPAP+quercetin	86.40 ± 2.33^c^	-24.44	91.18 ± 2.22^bc^	39.95	31.16 ± 0.72^b^	49.73	182.40 ± 1.12^b^	7.59	43.13 ± 1.27^b^	26.66

Data are expressed as mean ± SEM. The number of animals in each group is 6. ^a^Significant at *P* < 0.05 in comparison with the normal values. ^b^Significant at *P* < 0.05 in comparison with NAPAP values. ^c^Significant at *P* < 0.05 in comparison with NAPAP+MPHE values. Percentage changes are calculated by comparing NAPAP-administered control with normal control and NAPAP-administered treated rats with NAPAP-administered control.

**Table 6:** Effect of MPHE, hesperidin, and quercetin on kidney content of GSH and activities of GPx, GST, and SOD activities as well as LPO level of NAPAP-administered rats.

Parameter groups	LPO (nmol/100 mg tissue)	% change	SOD (U/g tissue)	% change	GSH (nmol/100 mg tissue)	% change	GPx (mU/100 mg tissue)	% change	GST (U/100 mg tissue)	% change
Normal	69.61 ± 1.72		99.73 ± 2.25		24.95 ± 0.56		154.78 ± 1.27		110.75 ± 1.73	
NAPAP	106.75 ± 1.23^a^	53.35	78.43 ± 3.54^a^	-21.35	17.00 ± 0.46^a^	-31.86	144.55 ± 1.10^a^	-6.60	90.73 ± 2.35^a^	-18.07
NAPAP+MPHE	78.95 ± 3.15^b^	-26.04	78.90 ± 5.55	0.59	22.70 ± 1.05^b^	33.52	151.15 ± 0.95^b^	4.56	102.81 ± 1.33^b^	13.31
NAPAP+hesperidin	86.21 ± 1.71^b^	-19.24	86.78 ± 7.25^b^	10.64	22.08 ± 1.33^b^	29.88	152.00 ± 1.27^b^	5.15	104.36 ± 1.53^b^	15.02
NAPAP+quercetin	80.15 ± 2.37^b^	-24.91	94.00 ± 4.00^b^	19.85	23.03 ± 0.97^b^	35.29	151.35 ± 0.62^b^	4.70	102.16 ± 1.45^b^	12.59

Data are expressed as mean ± SEM. The number of animals in each group is 6. ^a^Significant at *P* < 0.05 in comparison with the normal values. ^b^Significant at *P* < 0.05 in comparison with NAPAP values. Percentage changes are calculated by comparing NAPAP-administered control with normal control and NAPAP-administered treated rats with NAPAP-administered control.

RETRACTED

**Table 7:** Effect of MPHE, hesperidin, and quercetin on histopathological scores of livers of NAPAP-administered rats.

Histopathological changes	Score	Normal control	NAPAP	NAPAP+MPHE	NAPAP+hesperidin	NAPAP+quercetin
Inflammation	0	6 (100%)	—	2 (33.3%)	4 (66.7)	4 (66.7)
	I	—	1 (16.7%)	2 (33.3%)	2 (33.3%)	1 (16.7%)
	II	—	3 (50%)	2 (33.3%)	—	1 (16.7%)
	III	—	2 (33.3%)	—	—	—
Necrosis	0	6 (100%)	—	5 (83.3%)	2 (33.3%)	4 (66.7)
	I	—	1 (16.7%)	1 (16.7%)	2 (33.3%)	2 (33.3%)
	II	—	2 (33.3%)	—	1 (16.7%)	—
	III	—	3 (50%)	—	1 (16.7%)	—
Activated apoptosis	0	6 (100%)	—	3 (50%)	2 (33.3%)	5 (83.3%)
	I	—	1 (16.7%)	3 (50%)	4 (66.7)	1 (16.7%)
	II	—	4 (66.7)	—	—	—
	III	—	1 (16.7%)	—	—	—
Vacuolar degeneration	0	6 (100%)	—	2 (33.3%)	—	—
	I	—	1 (16.7%)	1 (16.7%)	1 (16.7%)	3 (50%)
	II	—	—	—	2 (33.3%)	3 (50%)
	III	—	5 (83.3%)	3 (50%)	3 (50%)	—
Vascular congestion	0	6 (100%)	—	3 (50%)	2 (33.3%)	4 (66.7%)
	I	—	2 (33.3%)	3 (50%)	3 (50%)	2 (33.3%)
	II	—	2 (33.3%)	—	1 (16.7%)	—
	III	—	2 (33.3%)	—	—	—
Stimulated Kupffer cell proliferation	0	6 (100%)	—	3 (15.0%)	1 (16.7%)	3 (15.0%)
	I	—	—	1 (16.7%)	2 (33.3%)	3 (15.0%)
	II	—	2 (33.3%)	2 (33.3%)	2 (33.3%)	—
	III	—	4 (66.7%)	—	1 (16.7%)	—

0: null; I: mild; II: moderate; III: severe lesions. The number of animals in each group is 6. The % in parentheses is the percent of animals in each grade of lesion.

**Table 8:** Effect of MPHE, hesperidin, and quercetin on histopathological scores of the kidneys of NAPAP-administered rats.

Histopathological changes	Score	Normal control	NAPAP	NAPAP+MPHE	NAPAP+hesperidin	NAPAP+quercetin
Inflammation	0	6 (100%)	—	5 (83.3%)	4 (66.7)	5 (83.3%)
	I	—	1 (16.7%)	1 (16.7%)	1 (16.7%)	1 (16.7%)
	II	—	2 (33.3%)	—	1 (16.7%)	—
	III	—	3 (50%)	—	—	—
Necrosis	0	6 (100%)	—	6 (100%)	5 (83.3%)	6 (100%)
	I	—	1 (16.7%)	—	1 (16.7%)	—
	II	—	1 (16.7%)	—	—	—
	III	—	4 (66.7)	—	—	—
Activated apoptosis	0	6 (100%)	1 (16.7%)	6 (100%)	5 (83.3%)	6 (100%)
	I	—	5 (83.3%)	—	1 (16.7%)	—
	II	—	—	—	—	—
	III	—	—	—	—	—
Congestion of renal blood vessels	0	6 (100%)	—	6 (100%)	4 (66.7%)	4 (66.7%)
	I	—	—	—	2 (33.3%)	2 (33.3%)
	II	—	2 (33.3%)	—	—	—
	III	—	4 (66.7)	—	—	—

0: null; I: mild; II: moderate; III: severe lesions. The number of examined sections in each group is six. The % in parentheses is the percent of animals in each grade of lesion.

## Data Availability

The data are available from the corresponding author upon reasonable request.

## Abbreviations

AC: Apoptotic cell
ALAT: Alanine aminotransferase
AP: Alkaline phosphatase
ASAT: Aspartate aminotransferase
Ca^2+^: Calcium ion
CMC: Carboxymethylcellulose
CYP2E1: Cytochrome P450 family 2 subfamily E member 1
CYP450: Cytochrome P450
dist. water: Distilled water
GPx: Glutathione peroxidase
GSH: Glutathione
GST: Glutathione-*S*-transferase
H&E: Hematoxylin and eosin
IL-4: Interleukin-4
LDH: Lactate dehydrogenase
LPO: Lipid peroxidation
MDA: Malondialdehyde
MPHE: Mandarin (*Citrus reticulata* L.) fruit peel hydroethanolic extract
NAD^+^: Nicotinamide adenine dinucleotide (oxidized form)
NADH: Nicotinamide adenine dinucleotide (reduced form)
NAPAP: N-Acetyl-para-aminophenol
NAPQI: N-Acetyl-*P*-benzoquinone imine
NRC: National Research Center
p53: Proapoptotic protein 53
PVDF: Polyvinylidene difluoride
RIPA: Radioimmunoprecipitation assay
ROS: Reactive oxygen species
rpm: Round per min
SDS-PAGE: Sodium dodecyl sulfate-polyacrylamide gel electrophoresis
SEM: Standard error of the mean
SOD: Superoxide dismutase
SPSS: Statistical Package for the Social Sciences
TBST: Tris-buffered saline with Tween 20
TNF-*α*: Tumor necrosis factor-*α*
*γ*GT: *γ*-Glutamyl transferase.
